# Bronchial epithelial and airway smooth muscle cell interactions in health and disease

**DOI:** 10.1016/j.heliyon.2023.e19976

**Published:** 2023-09-09

**Authors:** Reshed Abohalaka

**Affiliations:** Krefting Research Centre, Department of Internal Medicine and Clinical Nutrition, Institute of Medicine, Sahlgrenska Academy, University of Gothenburg, Gothenburg, Sweden

**Keywords:** Pulmonary disease, Airway, Asthma, COPD, Bronchial remodeling, Lung, Crosstalk

## Abstract

Chronic pulmonary diseases such as asthma, COPD, and Idiopathic pulmonary fibrosis are significant causes of mortality and morbidity worldwide. Currently, there is no radical treatment for many chronic pulmonary diseases, and the treatment options focus on relieving the symptoms and improving lung function. Therefore, efficient therapeutic agents are highly needed. Bronchial epithelial cells and airway smooth muscle cells and their crosstalk play a significant role in the pathogenesis of these diseases. Thus, targeting the interactions of these two cell types could open the door to a new generation of effective therapeutic options. However, the studies on how these two cell types interact and how their crosstalk adds up to respiratory diseases are not well established. With the rise of modern research tools and technology, such as lab-on-a-chip, organoids, co-culture techniques, and advanced immunofluorescence imaging, a substantial degree of evidence about these cell interactions emerged. Hence, this contribution aims to summarize the growing evidence of bronchial epithelial cells and airway smooth muscle cells crosstalk under normal and pathophysiological conditions. The review first discusses the impact of airway smooth muscle cells on the epithelium in inflammatory settings. Later, it examines the role of airway smooth muscle cells in the early development of bronchial epithelial cells and their recovery after injury. Then, it deliberates the effects of both healthy and stressed epithelial cells on airway smooth muscle cells, taking into account three themes; contraction, migration, and proliferation.

## List of Abbreviations

a-SMA: Alpha Smooth Muscle Actin
AEC: Alveolar Epithelial Cell
AECI: Alveolar Epithelial Cell Type I
AECII: Alveolar Epithelial Cell Type II
AHR: Airway Hyperresponsiveness
ASMC: Airway Smooth Muscle Cell
BEC: Bronchial Epithelial Cell
BNP: Brain Natriuretic Peptide
cAMP: Cyclic Adenosine Monophosphate
CCL: C–C Motif Chemokine Ligand
CCR: C–C Motif Chemokine Receptor
cGMP: Cyclic Guanosine Monophosphate
CLR: C-type Lectin Receptor
COPD: Chronic Obstructive Pulmonary Disease
COX-2: Cyclooxygenase-2
CSE: Cigarette Smoke Extract
CXCL: C-X-C Motif Chemokine Ligand
CXCR: C-X-C Motif Chemokine Receptor
ECM: Extracellular Matrix
EGF: Epidermal Growth Factor
FGF: Fibroblast Growth Factor
FoxP1: Forkhead Box P1
GABA: Gama-Aminobutyric Acid
GM-CSF: Granulocyte-Macrophage Colony-Stimulating Factor
HDM: House Dust Mites
IL: Interleukin
IP-10: IFN-γ-Induced Protein 10
IPF: Idiopathic Pulmonary Fibrosis
LTD4: Leukotriene D4
MCP: Monocyte Chemotactic Protein
MIP-1b: Macrophage Inflammatory Protein-1b
MMP: Matrix Metalloproteinase
NLR: Nucleotide-binding oligomerization domain-like Receptor
NO: Nitric Oxide
NOD: Nucleotide-binding Oligomerization Domain
PAR: Protease-Activated Receptor
PDGF: Platelet-Derived Growth Factor
PRR: Pattern Recognition Receptor
RV: Rhinovirus
TGF-β: Transforming Growth Factor Beta
TLR: Toll-Like Receptor
TNFα: Tumor Necrosis Factor Alpha
TRP: Transient Receptor Potential
TSLP: Thymic Stromal Lymphopoietin
VEGF: Vascular Endothelial Growth Factor

## 1 Introduction

Inflammatory respiratory diseases are a major public health concern with high rates of morbidity and mortality [1]. Among these diseases, asthma, with its various phenotypes, is a significant pulmonary disorder that affects over 300 million individuals worldwide, and its prevalence is rising notably in children and young adults [2]. Chronic Obstructive Pulmonary Disease (COPD) is another respiratory disease that causes progressive airflow restriction and is considered the third leading cause of death globally [3]. Additionally, less common chronic pulmonary diseases, such as Idiopathic Pulmonary Fibrosis (IPF), place a significant burden on the population, resulting in high mortality rates and treatment costs [4]. Unfortunately, radical cures for these diseases do not exist to date, and most current therapeutic strategies aim to suppress inflammation and promote bronchodilation. Therefore, comprehending the physiology of the respiratory system and the pathophysiology of these diseases is critical in developing future therapeutic approaches to treat or prevent these conditions.

### 1.1 Airway cellular pathophysiology

The airway in the respiratory system comprises several layers arranged in a specific manner to create a tube with a lumen (Fig. 1). The first layer, adjacent to the lumen, is a monolayer of cells known as the epithelium. The epithelial layer is a pseudostratified layer that encompasses numerous cell types, including ciliated cells, goblet cells that produce mucous, club cells, and basal cells. These cells are firmly attached to a basement membrane and to each other through tight junctions and adherens junctions. The basal membrane separates the epithelial layer from the subsequent layer, the lamina propria, which contains various immune cells and fibroblasts embedded in a mixture of extracellular matrix (ECM) mainly produced by the latter cells. The outermost layer around the lamina propria is formed by bands of airway smooth muscle cells [5], which are crucial in regulating broncho-motor tone and controlling the diameter of the airway [6].

**Fig. 1:** Adaptation of airway wall layers in response to stressful conditions, including inflammation, infection, and irritation from internal or external agents.

Each layer of the airway is comprised of a complex of different cell types that maintain lung homeostasis and protect the body against microbial and physical threats. Consequently, it is unsurprising that chronic lung diseases such as asthma, COPD, and pulmonary fibrosis arise due to the dysfunction of these cells and their interactions. Among these cells, bronchial epithelial cells (BECs) and airway smooth muscle cells (ASMCs) play a significant role in the pathogenesis of chronic lung diseases. For example, airway epithelial damage and abnormal repair, accompanied by an enlarged smooth muscle mass and increased cytokine production, are well-established characteristics of asthma [5,7,8]. In COPD, epithelial metaplasia and increased airway smooth muscle quantity correlate with airflow obstruction and, inversely, with lung function [9]. Moreover, epithelial cells play a pivotal role in initiating idiopathic pulmonary fibrosis and, alongside myofibroblasts, contribute to the disease's development [10,11]. Meanwhile, airway smooth muscle cells are linked to higher lung fibrosis and poorer clinical outcomes [12]. Therefore, it is essential to investigate the roles and interactions of BECs and ASMCs to reveal new therapeutic opportunities for many chronic respiratory diseases.

### 1.2 Advancements in cell-cell interactions research

For many years, researchers have explored the functions of bronchial epithelial cells and airway smooth muscle cells and their respective roles in respiratory diseases. Recently, however, there has been increasing attention towards the interactions between these two cell types and how they contribute to respiratory diseases [8]. This emerging interest is partly attributable to the development of modern, innovative research tools and models that have revealed new information on the communication and interaction between BECs and ASMCs in the development and progression of chronic respiratory diseases. A notable example of such advancements is the utilization of three-dimensional (3D) research tools, such as organoids, which consist of self-organized aggregates of single or multiple cell types cultivated within gels comprising a complex mixture of various extracellular matrix proteins. Through the implementation of organoids, researchers have gained insights into how different cell types interact with their surrounding microenvironment, mimicking *in vivo* conditions more accurately than traditional two-dimensional (2D) cell cultures. As a result, the co-culture of epithelial progenitor cells and mesenchymal cells utilizing this technique has yielded enhanced comprehension of their mutual interactions and the significance of their structural characteristics and topological arrangements in facilitating such interactions. The integration of three-dimensional (3D) cultures has significantly transformed biomedical research, thereby enabling enhanced investigations into organ development, disease modeling, and cell-cell interactions [[13], [14], [15], [16]].

Furthermore, a state-of-the-art approach that has emerged is the employment of organs-on-a-chip methodology, offering novel possibilities for presenting 3D cultured living cells under dynamic flow conditions. This technique permits the engineering of diverse tissue-tissue interfaces and 3D multicellular structures that closely resemble the functional units of human organs [17]. Notably, lung-on-a-chip and airway-on-a-chip models have gained widespread use in respiratory research. The focus of lung-on-a-chip studies has been particularly on establishing multilayered microfluidic devices that support the formation of differentiated airway epithelium, exhibiting phenotypes consistent with the ones found *in vivo*. These approaches not only provide an air-liquid interface for the cells but also facilitate a continuous flow of the culture medium, rendering the environment more physiologically relevant [[17], [18], [19], [20]].

Consequently, the findings derived from the studies using these novel research tools have contributed significantly to bolstering the evidence base concerning the interactions between BECs and ASMCs. However, despite these advancements, comprehensive reviews summarizing recent data on this subject remain scarce. This review aims to address this gap by providing an extensive overview of the expanding body of evidence concerning the interactions between BECs and ASMCs in the airways, along with their respective roles in chronic respiratory diseases. It is hoped that this contribution will facilitate future research planning and investigation. In order to foster a comprehensive understanding of this intricate subject, the review initiates by investigating the influence of airway smooth muscle cells on epithelial cells under both physiological and pathophysiological circumstances. Subsequently, it delves into a discussion regarding the implications of healthy and injured epithelial tissue on the contractility, migration, and proliferation of airway smooth muscle cells.

## 2 Influence of airway smooth muscles on epithelial cells

The significance of the airway smooth muscle (ASM) layer in healthy adult airways has been a topic of extensive deliberation among researchers [21]. However, the role of ASM in the pathophysiology of lung conditions and inflammatory diseases is well established. Indeed, ASM has been implicated in various lung conditions, including asthma, chronic obstructive pulmonary disease (COPD), and bronchiectasis.

The altered contractile function and mass of airway smooth muscle cells can lead to airway inflammation, hyperresponsiveness, and remodeling. Moreover, ASMC contractile activity is also modified in the context of lung fibrotic processes. These alterations are brought about by several pathways, including G-protein coupled receptor-based pathways, non-selective cation channels, particularly transient receptor potential channels (TRP), stretch-activated channels, Ca_2_+-dependent K+ channels, and store-operated calcium channels [6,22]. Damage to the epithelial layer can potentially trigger multiple changes regarding ion channels in ASMCs. The bronchial epithelial cells act as a barrier that separates ASMCs from the surrounding air. However, when ASMCs are exposed to hypotonic airway space liquid and gas due to airway epithelial cell barrier dysfunction, the activation of TRPV4 in ASMCs can trigger ASMC contraction. Additionally, damaged epithelial cells can cause a loss of ASMC constrictive capability in releasing NO, resulting in consistent airway contraction under hypotonic stimulation [23]. The phenomenon of heightened contractile response of airway smooth muscle, leading to excessive bronchoconstriction and airflow obstruction in response to relatively minor stimuli, is referred to as airway hyperresponsiveness (AHR). AHR holds significant implications in various respiratory conditions, notably in the context of asthma [24,25].

Furthermore, aside from their robust ability to constrict the airway lumen, ASMCs have the capacity to produce numerous proinflammatory growth factors, including transforming growth factor-β (TGF-beta), platelet-derived growth factor (PDGF), and fibroblast growth factor (FGF), as well as a wide range of cytokines, such as IL-1β, IL-5, IL-6, IL-8, and IL-17 [26]. Airway smooth muscle is capable of generating substantial quantities of extracellular matrix proteins, which can result in structural modifications in the airway [6]. Moreover, alterations in other ASMC functions, such as oxidant/antioxidant imbalances and metabolic dysfunctions, play a significant role in many pathophysiologies. For instance, abnormal mitochondrial function has been observed in ASMCs in patients with COPD, as evidenced by excessive reactive oxygen species production. This process serves as a secondary inducer of tissue inflammation and injury [6,27]. In addition, airway smooth muscle cells possess the capacity to transform from a contractile phenotype to a proliferative one, which can lead to heightened migration [28]. This transition in phenotype is associated with the downregulation of KCa_1.1_ channels and the upregulation of KCa_3.1_ channels [29]. This phenomenon is particularly noticeable under circumstances of stress, such as exposure to cigarette smoke and bacterial infection [30]. This shift in phenotype may contribute to the progression of airway remodeling in several chronic lung diseases. Airway remodeling encompasses pathological alterations, namely augmented airway smooth muscle mass, thickening of the basement membrane, and hyperplasia of mucus glands, as illustrated in Fig. 1. These prevalent attributes of COPD and asthma significantly contribute to the chronic hindrance of airflow observed in these diseases [31,32]. Therefore, understanding the underlying mechanisms and factors that contribute to this process is essential for the development of effective therapeutic strategies to combat these disorders. However, further investigations are necessary to identify additional factors that may be involved in the phenotypic transformation of ASMCs.

When airway smooth muscle cells are subjected to stressful conditions, they have the potential to exert an impact on epithelial cells. This interaction between airway smooth muscle cells and epithelial cells can have a significant effect on the functioning of the respiratory system. Specifically, stress-induced activation of airway smooth muscle cells may lead to the production of various cytokines and growth factors that can modulate epithelial cell behavior. In this context, Faiz et al. found that the secretion of CCL20 by ASMCs was increased by IL-1B in both healthy and asthmatic patients, although the effect was more pronounced in cells taken from asthmatic individuals. The release of CCL20 by ASMCs induced mucus production in BECs primarily by binding to CCR6 receptors on mucus-producing goblet cells in the epithelium [33]. This is a crucial consideration, particularly in light of the fact that the levels of IL-1B are markedly elevated during pulmonary infections. Thus, elucidating the role of IL-1B in the pathogenesis of pulmonary infections may have broader implications for the influence of infectious agents in chronic lung diseases.

Additionally, under certain conditions, ASMCs can impact the cytokine production of BECs. Deacon et al. reported that human ASMCs increased the secretion of amphiregulin in response to bradykinin exposure. This increase in amphiregulin levels directly contributed to the production of CXCL8, vascular endothelial growth factor (VEGF), and COX-2 in airway epithelial cells [8]. A recent study revealed that CCL20 released from human ASMCs significantly increased rhinovirus replication within the epithelium *in vitro*. This effect was mediated via the antiviral protein kinase RNA-activated (PKR) pathway, highlighting another dimension of ASMCs' impact on respiratory diseases, where frequent exacerbations due to respiratory viruses, such as asthma and chronic obstructive pulmonary disease, are often observed [34].

### 2.1 Role of epithelial-smooth muscle cell interactions during development

In comparison to the role of airway smooth muscle cells in adult life, their role in lung development is better understood. Numerous studies have demonstrated that ASMCs play a crucial role in the development of epithelia during organogenesis. During lung development, the lung starts as a simple epithelial tube surrounded by mesenchyme cells that eventually differentiate into several different cell types. Smooth muscle cells, which arise from fibroblast growth factor 10-expressing mesenchymal cells, are among these cell types [35,36].

The epithelium layer experiences branching morphogenesis to generate the conducting airways, such as bronchi and bronchioles [37]. However, epithelial proliferation alone is insufficient for branching, and the presence of smooth muscle wrapping is necessary to mold the epithelium into a tube-like shape [38]. This task is particularly crucial in the case of cartilage-lacking bronchioles, where smooth muscle cells are necessary for providing the required elasticity to maintain the patency of the airway [39]. These smooth muscle cells exert physical forces to shape the epithelia thanks to their contractile phenotype. Nevertheless, recent computational models have suggested that epithelial folding could be driven by the stiffness of the smooth muscle layer surrounding the epithelial cells rather than by contractile forces [40]. This hypothesis was also confirmed by Goodwine et al. in a recent study, where the authors demonstrated that the presence of smooth muscle cells alone was sufficient for airway branching morphogenesis in mice, even if these smooth muscle cells lacked the contractile phenotype [41]. Moreover, Palmer et al. showed that this stiffness acts as a mechanical wall against which fluid pressure pushes the epithelial cells during epithelial branching in the lizard lung. To illustrate this effect, the authors used the example of a stress ball, where the fluid pressure inside the developing tube pushes the epithelial cells against the holes of a meshwork of smooth muscle layer [42].

Similar outcomes were observed in 3D cell culture studies, such as the innovative method developed by Güney et al. [43]. In this study, airway epithelial cells were seeded inside an extracellular matrix (ECM)-mimicking structure of agarose and hydrogel (agrogel) and allowed to develop and proliferate for about three weeks. The authors reported that when seeded alone, the epithelial cells formed spheres inside the 3D structure of agrogel. However, adding stromal cells such as ASMCs increased the survival of the epithelial cells and, most importantly, transformed the spherical 3D structure into a tubule. The formation of the tubule was driven by the epithelial cells and was surrounded by stromal cells. Thus, the crosstalk between BECs and ASMCs was crucial for the branching of spheres into a tube-like structure, which the authors called bronchotubules.

In mice, the presence of SMA α-expressing smooth muscle cells adjacent to the airway epithelium prior to epithelial branching in embryonic mouse lungs is crucial. The localized presence of these smooth muscle cells is necessary for epithelium branching, as the surgical removal of smooth muscle entirely abolished branching [35]. Goodwin et al. also discovered that during mouse lung development, epithelial proliferation alone is inadequate for the generation of domain branches. Instead, smooth muscle wrapping is necessary to shape the epithelium into a branch [38]. Following epithelium branching, fibroblast growth factor 10-expressing cells move proximally along the airway and express smooth muscle-specific genes, such as α-actin-2 [44]. These cells also release fibroblast growth factor 10, which acts on the epithelial progenitors to prevent differentiation and promote proliferation [45]. Any abnormalities in airway smooth muscle cells during mouse lung development are associated with a distinct epithelial phenotype characterized by reduced basal cell number, precocious club cell differentiation, and increased secretoglobin expression [39]. Even after lung development, Volckaert et al. reported that the embryonic fibroblast growth factor 10 signaling pathway is reactivated in mature ASMCs following bronchial epithelial cell injury in adult mouse lungs. This action allows ASMCs to create an airway epithelial stem cell niche that aids in BEC repair [45]. In this regard, Moiseenko et al. discovered that this BEC-repair supporting ASMC population is distinct from pre-existing airway smooth muscle cells and is critical for renewing BECs in the adult lung [46]. Nevertheless, in a recently published study, Young et al. reported that the differentiation of airway smooth muscle during lung development is not required for lung branching morphogenesis in mice. Nonetheless, it is vital for establishing airway size and tracheal cartilage segmentation [47].

At first glance, it may seem unimportant to comprehend the interplay between airway smooth muscle cells and bronchial epithelial cells during organ development for the purpose of developing new treatment strategies for lung diseases. However, it is crucial to understand these interactions for organ engineering and the development of innovative 3D *ex vivo* models, such as organoids and lung-on-a-chip, which can help in the testing and development of new potential medications. These advanced models are of great significance because they provide a 3D structure that accurately mimics the lung microenvironment and the organ's complexity, enabling cells to interact with the surrounding extracellular matrix and external environment while retaining close interaction with each other [37,48]. These models are therefore useful tools for investigating cellular mechanisms, drug screening, and personalized medicine and may ultimately lead to the discovery of more effective treatments for various lung diseases. Therefore, understanding the interaction between airway smooth muscle cells and bronchial epithelial cells during organ development is a critical step in the development of these models and the advancement of lung disease research.

## 3 Epithelial influence on airway smooth muscle cells

Airway epithelial cells, characterized by their tight junctions, constitute the initial line of defense against various pollutants and pathogens in the lungs. Moreover, they play a pivotal role in the airway clearance system, which encompasses secreted mucus, ciliary beating, and antimicrobial peptides. Historically, it was widely assumed that the primary function of epithelial cells was to act as a mechanical barrier against inhaled foreign particles [49]. However, recent advancements in research techniques have enabled a deeper investigation into the interactions of epithelial cells with other cellular components, revealing a more intricate and multifaceted role in both normal and pathophysiological conditions. Therefore, in contemporary times, there exists widespread acceptance regarding the notion that the epithelium serves a purpose that extends beyond its mere physical structure.

The cellular composition and function of epithelial cells vary across different regions of the airways. The proximal airways predominantly consist of bronchial ciliated epithelial cells, whereas the distal alveolar region comprises alveolar epithelial cells (AECs). AECs can be further classified into two distinct subtypes: type I and type II. Type I cells (AECI) predominate the alveolar surface and are well-suited for facilitating gas exchange, while type II cells (AECII) are responsible for producing and secreting pulmonary surfactant to prevent alveolar collapse and improving lung compliance [50,51]. In addition, epithelial cells possess a range of pattern recognition receptors (PRRs), including toll-like receptors (TLRs), nucleotide-binding oligomerization domain (NOD)-like receptors (NLRs), C-type lectin receptors (CLRs), and protease-activated receptors (PARs), allowing them to recognize various foreign particles [49]. Furthermore, bronchial epithelial cells can secrete an array of chemokines and cytokines, such as interleukin-1 beta (IL-1β), interleukin-6 (IL-6), interleukin-25 (IL-25), interleukin-33 (IL-33), C-X-C motif chemokine ligand 8 (CXCL8), C–C motif chemokine ligands (CCL5, CCL17, and CCL20), granulocyte-macrophage colony-stimulating factor (GM-CSF), and thymic stromal lymphopoietin (TSLP), which recruit and activate various cell types and phenotypes [49,52,53].

Due to their location, pulmonary epithelial cells are highly vulnerable to injury. This is primarily due to their constant exposure to a range of exogenous stressors, such as bacterial and viral insults, cigarette smoke, and airborne pollutants, as well as endogenous signals, such as oxidative stress. In response to injury, these cells typically coordinate the immune response, aid in the removal of invading pathogens, and promote tissue homeostasis. Nevertheless, in numerous chronic lung diseases, this regulatory process becomes disrupted, resulting in persistent inflammation and the remodeling of functional tissue structure into a dysfunctional one [51].

In a healthy airway, the lamina propria layer serves to separate the epithelial sheet from the smooth muscle layer, thereby precluding direct contact between the epithelial and airway smooth muscle cells. The diffusion of soluble mediators through the lamina propria layer is therefore required for the epithelium to exert an effect on ASMCs [54]. When confronted with air pollutants or environmental pathogens, the epithelium can release such mediators, resulting in airway narrowing, obstruction, and exacerbation in individuals with asthma and COPD [7]. Consequently, targeting these paracrine signals from the airway epithelium to the underlying smooth muscle layer has the potential to serve as a promising approach for developing novel treatment strategies for asthma, COPD, and other chronic pulmonary diseases [55]. In addition, recent studies suggest that the epithelium layer can also influence ASMCs under normal conditions. Hereafter, perhaps these new strategies could prevent the development of the disease and the structural remodeling accompanying them. The epithelial cells in the airway tend to have different and complex effects on ASMCs. Depending on the outcome of these effects, the review will categorize them into three main themes: Effects that impact ASMC contractility, actions that affect ASMC migration, and interactions that alter ASMC proliferation.

### 3.1 Epithelial influence on airway smooth muscle cell contractility

Since the mid-1980s, researchers have endeavored to comprehend the impact of the airway epithelium on airway smooth muscle tone. The initial investigation, which utilized canine and dog bronchi, demonstrated *in vitro* that the removal of the epithelium increased the sensitivity of airway smooth muscle to various constricting agonists [56]. Subsequently, many researchers verified this phenomenon, along with reporting that the removal of the epithelium reduced airway smooth muscle responsiveness to some relaxing agents using *in vitro* cattle, guinea pigs, and rabbit trachea [57]. However, it is currently well-established that prostaglandins and nitric oxide released from the epithelium are responsible for this effect, and these studies were previously reviewed [[56], [57], [58]]. Therefore, the aim of this review is to concentrate on the emerging new data on the effects of the epithelium on ASMCs outside the prostaglandins and leukotrienes pathways, outlining the novel probable paths and outcomes of research studies that use innovative research models to achieve this purpose.

The epithelium plays a multifaceted role in influencing airway smooth muscle cells under normal and pathophysiological conditions. While the prostaglandins pathway has been shown to impact ASMCs, recent data indicate that other pathways are involved as well. Although these pathways operate through different mechanisms, existing literature suggests that the epithelium is likely involved in promoting ASMC relaxation under normal conditions but contributing to hyperresponsiveness in stressful environments (as depicted in Fig. 1, which shows adaptation of the airway wall layers to stressful settings).

1. The Impact of Epithelium on Airway Smooth Muscle Cell Relaxation:

The airway epithelium serves as the primary endogenous source of γ-aminobutyric acid (GABA) in the airways of mice, humans, and guinea pigs [[59], [60], [61]]. Gallos et al. [59] reported that GABA released from the epithelium contributes to both *in vitro* and *in vivo* relaxation of ASMCs. Gabazine, a GABA receptor antagonist, has been shown to augment the ASMC response to acetylcholine in healthy human airway tissue and guinea pig trachea. Likewise, targeting the GABA receptor in the epithelium in mice studies led to reduced ASMC contraction. However, this pharmacological approach yielded contradictory effects on mucus production in murine allergic asthma models, where GABA receptor agonists reduced mucus production in one study [61] while GABA receptor antagonists had a similar effect in another study [60]. Hence, further investigations are warranted to assess the viability of targeting the GABA receptor in the epithelium as a potential treatment for diseases exhibiting features of airway hyperresponsiveness, such as allergic asthma.

Brain natriuretic peptide (BNP) is an endogenous hormone secreted primarily by the ventricular myocardium under normal conditions and elevated in heart failure [62], but not in asthma and COPD patients [63]. Calzetta et al. reported that BNP increased the levels of acetylcholine and nitric oxide in the supernatant of BECs when added to the cell culture. Remarkably, the acetylcholine-high supernatant of BECs contributed to ASMCs relaxation in cell culture. To explain the pro-relaxant effect of the previously mentioned supernatant in the study, the authors investigated the role of the muscarinic M2 receptor. As the selective blocking of this receptor demolished this effect, the authors suggested that the substance discharged from BECs enhances the second messenger cyclic guanosine monophosphate (cGMP) concentration inside ASMCs, acting specifically on the muscarinic M2 receptor [64]. Moreover, the administration of B-type natriuretic peptide (BNP) resulted in a notable increase in peak expiratory flow rate (PEFR) in patients experiencing acute asthma exacerbations, with no significant occurrence of adverse effects. This suggests that BNP may hold promise as a potential therapeutic intervention, especially for individuals exhibiting varied responses to B2 receptor agonists [65]. As a result, the potential bronchodilator role of BNP in safeguarding against airway hyperresponsiveness in asthma, through the interactions between BECs and ASMC, as previously suggested [66], becomes more evident.

In another study, the supernatant of healthy unstressed human BECs and commercial epithelial cell line BEAS-2B contributed to the relaxation of ASMCs when added to ASMCs culture. Further, the supernatant of unstimulated BECs altered the contractile phenotype of ASMCs. This alteration was characterized by downregulating α-smooth muscle actin (α-SMA) in ASMCs. Furthermore, the new phenotype expressed higher cyclic adenosine monophosphate (cAMP) in response to constricting agonists such as histamine [67].

2. Epithelial Cell-Mediated Modulation of Airway Smooth Muscle Cell Contraction:

On the contrary, bronchial epithelial cells have been observed to amplify the contractile response of ASMCs under stressful and tense conditions, as opposed to their usual role of promoting relaxation under normal conditions. Such conditions may arise from either endogenous or exogenous stimuli, or from internal or external stressors. For example, *in vitro* experiments have shown that the supernatant of mechanically compressed human BECs increases the contraction of ASMCs in response to histamine [68]. Given that BECs are subjected to significant mechanical compression during acute bronchoconstriction, the findings of Lan et al. highlight the importance of targeting the influence of BECs on ASMCs as a potential therapeutic strategy for bronchodilator-resistant airway diseases. The authors also reported that this effect was dependent on endothelin-1, as blocking endothelin receptors in ASMCs eliminated this observation. In addition, Zhou et al. [69] used an *ex vivo* lung slice model in rats to demonstrate that physical injury to BECs was responsible for the contraction of ASMCs. Furthermore, even the rupture of a single epithelial cell induced rapid and widespread airway constriction by triggering a distinct instantaneous calcium wave in the epithelium and multiple waves in ASMCs. The authors therefore suggested that the physical stress of BECs may lead to the release of soluble mediators from the epithelium into the smooth muscle layer. The validation of the modulation effect exerted by physically injured epithelial cells on ASMCs necessitates further investigation through *in vivo* studies. Nevertheless, it is plausible that this phenomenon might instigate a feedback loop, partially contributing to the observed bronchodilator resistance in certain asthma and COPD patients [[70], [71], [72]].

Inflammatory stressors, such as infection, have been demonstrated to contribute to the constriction of BECs on ASMCs. Among these stressors, rhinovirus (RV) is one of the most commonly encountered infections in both pediatric and adult respiratory systems [73,74]. RV infection has been associated with a heightened risk of asthma in children and exacerbations in adult asthmatics. Thus, the use of RV in research and disease models for asthma has become increasingly widespread, given its clinical relevance and potential to elucidate the underlying mechanisms of this disease [73]. Parikh et al. conducted a study that aimed to investigate the relationship between rhinovirus (RV) infection and airway hyperresponsiveness (AHR) using an *ex vivo* human model of asthma. The study demonstrated that RV infection of the epithelium led to the induction of AHR. The authors found that this induction was associated with increased responses of ASMCs to carbachol and an increased influx of intercellular calcium [75]. Additionally, the authors examined the effect of RV infection on BECs. The infected epithelial cells expressed higher levels of IFN-γ-induced protein 10 (IP-10) and macrophage inflammatory protein-1b (MIP-1b). It is worth mentioning that the findings of the study have important implications for our understanding of the pathogenesis of AHR in asthma, as the authors observed that RV infection did not increase the release of cytokines typically known to cause AHR, such as IL-13 and IL-33, from the infected epithelial cells. In point of fact, cytokine IL-13 has been shown to have the capability of inducing AHR even in the absence of direct effects on ASMCs. This observation was demonstrated by Kuperman and colleagues, who utilized genetically modified mice that only expressed functional IL-13 receptors in the BECs while lacking expression in ASMCs. The study by Kuperman et al. elucidated that cytokine IL-13 instigated BECs to enhance the response of ASMCs towards agonists, thus elucidating the molecular mechanisms underlying AHR induction [76].

β2-Adrenoreceptor agonists are commonly used as effective bronchodilators in asthma. However, recent studies have suggested that activation of the β2 adrenoreceptor–β arrestin pathway can produce contradictory effects in murine asthmatic models. In a study similar to the aforementioned research, P. Nguyen et al. [77] genetically modified mice to express β2-adrenoreceptors only in their epithelial cells. Using IL-13 as a stressor, the authors observed the classical effects of IL-13 on the airways, such as airway hyperresponsiveness, eosinophilic inflammation, and mucus production. Moreover, the study demonstrated that blocking β2-adrenoreceptors in the epithelial cells eradicated all previously mentioned effects of IL-13, while stimulating β2-adrenoreceptors exacerbated these effects. Hence, the authors concluded that the activation of the β arrestin pathway in BECs is responsible for these outcomes, independently of the direct pathway actions in ASMCs. However, the authors did not identify the exact mechanism by which BECs influence ASMCs contraction. Nonetheless, they suggested that cytokines released from BECs towards ASMCs, particularly the production of CCL2, CCL24, and CXCL1, significantly increased following exposure to IL-13.

In the absence of tense and stressful conditions, the impact of BECs on ASMCs may also be attributed to genetic factors. Li et al. [55] have reported that specific phenotypes of murine epithelium, which lack the transcription factors forkhead box P1 and P4 (Foxp1 and Foxp4), can elicit AHR and ASMC contractility. Notably, the authors have highlighted that the loss of Foxp1 and Foxp4 expression results in the secretion of neuropeptide Y from the epithelial cells. This powerful vasoconstrictor peptide increases Rho kinase activity and thereby phosphorylates the myosin light chains in ASMCs, without altering the inflammatory profile or cytokine levels. These findings could have important implications for understanding the underlying mechanisms involved in the development of respiratory disorders such as asthma. It also highlights the importance of exploring the genetic factors involved in the development of these disorders and the potential role of neuropeptide Y as a therapeutic target for the treatment of asthma.

The airway's epithelial cells play a crucial role as the first line of defense against harmful microorganisms and environmental stressors. In light of this, restricting their access to the airways is imperative. Thus, it is logical to consider influencing the airway smooth muscle cells to act inversely in standard and acute settings to limit the access of these stressors (Fig. 2 summarizes the effect of bronchial epithelial cells on airway smooth muscle contractility). Nonetheless, malfunctioning of this tightly controlled airway regulation may lead to pathophysiological conditions. Therefore, gaining a better understanding of the impact of bronchial epithelial cells on airway smooth muscle contractility could facilitate the development of novel therapeutic strategies for respiratory illnesses. These therapeutic options could be particularly significant for patients with abnormal resistance to typical bronchodilators.

**Fig. 2:** Contradictory effects of bronchial epithelial cells on airway smooth muscle contractility.

Influence of Epithelium on the Migration of Airway Smooth Muscle Cells:

Airway remodeling is a constellation of chronic alterations in the structure of the airways that can be observed in several respiratory diseases. This constellation encompasses various observations, including epithelial injury, insufficient recovery, heightened airway wall thickness, and increased airway smooth muscle cell mass [78]. For an extended period of time, researchers believed that hypertrophy and hyperplasia of airway smooth muscle cells were the primary factors causing the increased wall thickness and airway smooth muscle cell mass. However, recent studies suggest that the migration of airway smooth muscle cells may also play a role in the augmentation of airway smooth muscle cell mass, particularly in individuals suffering from asthma [79]. These recent findings are promising in revealing new insights into the complex mechanisms that contribute to airway remodeling.

In recent years, there has been a growing interest in the *in vitro* investigation of two distinct types of co-culture that involve BECs and ASMCs. Direct co-culture refers to a situation where the cells share a culture and are in direct contact with one another, whereas indirect co-culture involves the separation of the cells physically, but they share the same culture medium [80]. Alongside the development of novel techniques and migration assay tools in cell culture models [80], research has started to unravel the potential impact of BECs on the migration of ASMCs. As of the present, the comprehensive understanding of how the epithelium influences ASMC migration under normal conditions remains incomplete. Nonetheless, numerous studies have consistently demonstrated that the impact of BEC on ASMC migration is minimal in healthy conditions [79,81,82]. However, it is worth noting that several endogenous and exogenous stressors play an essential role in activating BECs to enhance the migration of ASMCs in cell culture.

1. Impact of Endogenous Stressors on the Modulation of BECs-induced ASMCs Migration:

YKL-40 is a glycoprotein that is expressed and secreted by various cell types in humans. Elevated serum levels of YKL-40 have been linked to respiratory diseases such as asthma and COPD [81]. Consequently, YKL-40 has been proposed as a potential biomarker for identifying COPD and the medication-resistant T2-low phenotype of asthma [83,84]. Several studies have indirectly linked YKL-40 to increased migration of human ASMCs through its effects on BECs. For instance, Tang et al. [81] found that YKL-40 increases the expression and production of IL-8 by human BECs and BEAS-2B epithelial cell lines in a dose-dependent manner. This effect is dependent on MAPK and NF-κB pathways, as blocking either pathway attenuates the amplified chemokine levels. When the researchers treated ASMCs with the supernatant of these epithelial cells, they observed that increased levels of IL-8 were the primary contributor to the increased migration of human ASMCs *in vitro*. Furthermore, depletion of IL-8 from the cell culture medium abolished this effect. It should be noted that YKL-40 can directly enhance ASMC migration, independent of the contribution of BECs. In this regard, Bara et al. [82] reported that YKL-40 increased ASMC migration *in vitro* without affecting the cytokine production profile of ASMCs. However, higher expression of YKL-40 in the epithelial cells of asthmatic patients was positively correlated with greater ASMC mass. Hence, additional research is imperative to elucidate whether the effects of BECs on ASMC migration arise from the direct influence of the released YKL-40 from BECs or if it is attributed to the impact of IL-8, which is released from BECs in response to the elevated YKL-40 levels.

Tumor necrosis factor alpha (TNFα) is an endogenous mediator and a pro-inflammatory cytokine that exerts indirect implications on amplified migration of ASMCs and induces the recruitment of neutrophils and eosinophils in asthma and COPD [[85], [86], [87]]. Studies have shown that when the supernatants of both the BEAS-2B epithelial cell line and human bronchial epithelial cells were exposed to TNFα in cell culture for 24 h, higher levels of IL-8 and RANTES (CCL5) were expressed in a concentration-dependent manner, while lower levels of TGF-β were observed. The increased expression of these two chemokines resulted in the direct increase of ASMC migration, as demonstrated by the Boyden chamber analysis. In addition, blocking one of these chemokines decreased the migration of ASMCs in cell culture [79]. These findings suggest that TNFα-induced expression of IL-8 and CCL5 in BECs may play a role in the pathogenesis of asthma by promoting ASMC migration. The significance of this phenomenon is heightened when considering the frequent elevation of TNFα levels in various inflammatory respiratory diseases, as well as in recurrent viral and bacterial infections. Therefore, there is a compelling need for a comprehensive investigation and understanding of the mechanisms underlying TNFα dysregulation. Such an investigation holds the potential to provide valuable insights into the short-term and long-term development and progression of these pathologies. For instance, it may elucidate the mechanisms behind airway remodeling observed in patients with asthma and COPD [88,89]. Moreover, targeting TNFα could offer a promising approach to preventive treatment strategies in these contexts.

2. Impact of Exogenous Stressors on the Modulation of BECs-induced ASMCs Migration:

The respiratory system is the primary interface for interactions between the body and the external environment, particularly the epithelium. This epithelial layer is continuously exposed to various exogenous factors, including microorganisms, pollutants, and allergens, which have been found to trigger or exacerbate chronic respiratory diseases. For instance, cigarette smoking has been identified as a critical risk factor for chronic obstructive pulmonary disease [90], while second-hand smoke exposure also contributes to the development of this condition [91]. Moreover, rhinovirus has been associated with asthma development and COPD exacerbations [9,73]. Importantly, it has been observed that certain exogenous factors can stimulate the migration of ASMCs by acting on BECs. Recent studies have shown that cigarette smoke extract can enhance the production of interleukin-8 (IL-8) and transforming growth factor-beta (TGF-β) by human epithelial cell lines, such as A549, in cell culture [92]. These cytokines, in turn, increase the migration of ASMCs when they are present in the cell culture. Blocking either IL-8 or TGF-β significantly inhibits the migration of ASMCs toward cigarette smoke-exposed epithelial cells. Moreover, the impact of epithelial cells on ASMC migration can be further intensified by the presence of muscarinic agonists such as carbachol. This effect is mediated through the activation of the M3 receptor on the bronchial epithelial cells [92]. Hence, the interactions between BECs and ASMCs, encompassing pathways governed by IL-8 and TGF-β cytokines, alongside the involvement of the M3 muscarinic receptor, hold significant relevance in the context of both regular management and prophylactic interventions for COPD patients and the broader population of smokers.

Nonylphenol, another environmental pollutant with estrogen-like activities, augmented the production of IL-6 and IL-8, but not CCL5, from HBE135-E6E7 and BEAS-2B human epithelial cell lines in cell culture. Although nonylphenol increased the apoptosis of these cell lines, the conditional medium created from the supernatant of these cells significantly increased the migration of ASMCs *in vitro*. This effect depended on both IL-6 and IL-8, as depleting either from the conditioned medium altered the migration amplification [93].

With regards to exogenous factors, the supernatant of human bronchial epithelial cells was found to induce migration of human asthmatic airway smooth muscle cells in indirect co-culture after being infected with rhinovirus. This increased migration was associated with higher production of the chemokines CXCL10, CXCL8, and CCL5 from BECs. Interestingly, depletion of only CCL5 from the supernatant of BECs was sufficient to prevent the migration of ASMCs, thereby suggesting that CCL5 plays a vital role in ASMC migration. The authors also observed that even though ASMCs highly express the CXCR3 receptor, its natural ligand CXCL10 had a lesser impact on the increased migration of ASMCs. However, ASMCs also expressed CCR1, CCR3, and CCR5 receptors to a lesser extent, which suggests that the effect of CCL5 on ASMC migration could be mediated through one of these receptors. Notably, the authors used an anti-CCL5 antibody, instead of receptor blockage, to investigate the impact of CCL5, which makes it difficult to draw a more robust conclusion [94]. Additionally, in line with the previous study, human BECs were found to increase the migration of human asthmatic ASMCs, but not healthy ASMCs, in indirect co-culture after being infected with rhinovirus. The authors reported that this outcome was associated with the higher production of CXCL10 and CXCL9. Furthermore, they found that CXCR3 antibodies could block this effect, thereby suggesting that CXCL10 drives this specific migration by activating CXCR3. Interestingly, Celle et al. reported that the distance between the basal membrane of epithelial cells and the smooth muscle layer in the airways of asthmatic patients was shorter compared to healthy subjects [95].

In brief, several studies have shown that IL-8 (CXCL8), CXCL10, and RANTES (CCL5) have a positive impact on the migration of smooth muscle cells in the airways. This is of great significance, particularly given that BECs can generate all of these cytokines in response to a stressful environment, particularly in individuals with asthma. These cytokines could potentially play a significant role in reducing the distance between the epithelial and smooth muscle layers, which is a hallmark of airway remodeling. However, to make more definitive statements about the role of these cytokines, further studies and investigations are required. Nonetheless, CXCL8, CXCL10, and CCL5, along with their corresponding receptors (CXCR1 and CXCR2), CXCR3, and CCR5, respectively [96,97], appear to be a promising therapeutic target for preventing ASMC migration in bronchial remodeling and, as a result, exacerbation of the disease in patients with chronic lung conditions, such as asthma and COPD.

### 3.2 Effects of epithelial factors on the proliferation of airway smooth muscle cells

The thickening of the smooth muscle layer in the airway wall is among the most significant characteristics of bronchial remodeling. Moreover, numerous studies have linked increased smooth muscle mass to asthma severity in both adults and children [98]. Consequently, novel asthma treatments such as bronchial thermoplasty aim to target the smooth muscle cells of the airway. Additionally, although most of the traditional therapies for asthma and chronic obstructive pulmonary disease are geared towards bronchodilation and suppressing the activation and infiltration of inflammatory cells into the airways [99], these medications are also considered potent inhibitors of airway smooth muscle cell proliferation.

The effects of the epithelium on ASMC proliferation are more intricate than their influence on migration and contraction. Numerous studies have shown that relaxed and stressed bronchial epithelial cells increase the proliferation of ASMCs in both *in vitro* and *in vivo* settings. Indirect co-culture of healthy human BECs and BEAS-2B cell lines with human ASMCs led to a shift in the phenotype of the latter cells towards a proliferative phenotype. Consequently, ASMCs downregulated a-smooth muscle actin (a-SMA) and myocardin and expressed lower intracellular calcium and higher cAMP levels in response to histamine [67]. Furthermore, Malavie et al. have reported that the direct co-culture of unstimulated and healthy human BECs with human ASMCs increased the proliferation index of ASMCs *in vitro*. The co-culture supernatant showed higher levels of IL-6, IL-8, monocyte chemotactic protein (MCP-1), and matrix metalloproteinase (MMP-9) than only ASMCs culture, and all of the aforementioned mediators correlated with the degree of ASMC proliferation. The increased proliferation index of human ASMCs in co-culture was decreased by inhibiting IL-6 and/or IL-8 and abolished by inhibiting MCP-1 and/or MMP-9 pathways. Notwithstanding, physically injured human BECs have been shown to increase the proliferation index of human ASMCs *in vitro* even more than healthy BECs, and the co-culture expressed even higher concentrations of IL-6, IL-8, MCP-1, and MMP-9. However, when comparing the injured and healthy BECs cultures, only the production of MMP-9 tends to increase between the wounded and uninjured epithelial cells. These findings suggest that injury-induced MMP-9 release by epithelial cells is vital in the proliferation of ASMCs [54]. Moreover, since mechanical compression also increased BECs-induced ASMC proliferation, BECs-ASMCs interactions play a fundamental role in how bronchoconstriction contributes to bronchial remodeling [68]. Studies conducted *in vivo* have yielded similar findings, where mechanical injury to the epithelial layer of rabbit trachea has stimulated proliferation in the airway smooth muscle layer.

It should be noted that physical injury or compression is not the only factor that can induce the proliferation of ASMCs by BECs. Many exogenous and endogenous stressors can also produce this effect. Tang et al. demonstrated that both human BECs and BEAS-2B cells increased the proliferation of human ASMCs *in vitro* when exposed to YKL-40. This exposure resulted in an increase in the production of the cytokine IL-8 (CXCL8) by BECs [81]. Additionally, YKL-40 directly increased the proliferation of ASMCs in cell culture, even in the absence of BECs, by activating the PAR-2-receptor signal [82]. Regarding endogenous stimulators, amphiregulin, a member of the epidermal growth factor (EGF) family, is a potent growth stimulator. Amphiregulin has been shown to encourage BECs to increase growth factor expression in ASMCs mainly by acting on the COX-2 enzyme of BECs [8]. Furthermore, leukotriene D4 induced BECs to increase the production of TGF-β1 in cell culture. The TGF-β1-rich supernatant of BECs significantly increased the proliferation of ASMCs *in vitro* [100]. As LTD4 can increase TGF-β1 production from BECs by acting on cys-LT receptor 1 (CysLT1), the authors hypothesized that a paracrine loop of TGF-β1 secretion from BECs and ASMCs could be involved in ASMC proliferation *in vivo* as well. It is clear that a range of factors can contribute to the proliferation of ASMCs by BECs, including physical and chemical stressors, such as YKL-40, amphiregulin, and leukotriene D4. These findings highlight the importance of investigating the molecular mechanisms underlying ASMC proliferation in response to BEC stimulation, which may lead to the development of novel therapeutic approaches to prevent and treat airway remodeling in chronic lung conditions.

Respiratory inflammatory conditions, including asthma and COPD, are recognized for their recurrent exacerbations, which are mainly triggered by exogenous factors or stimuli such as bacteria, cigarette smoke, house dust mites (HDM), and other allergens [91,[101], [102], [103]]. Lu et al. demonstrated that human alveolar epithelial cells exposed to cigarette smoke extract (CSE) enhanced the ability of human airway smooth muscle cells to repair injury [92]. Furthermore, epithelial cell stimulation by house dust mite extract was found to increase asthmatic ASMC proliferation, but not that of non-asthmatic subjects, through a protease-activated receptor (PAR)-2-dependent epithelial production of leukotrienes C4. Moreover, asthmatic ASMCs were observed to overexpress leukotriene receptor CysLT1 [103]. Additionally, the environmental pollutant Nonylphenol was found to increase the production of IL-6 and IL-8 by human bronchial epithelial cells and BEAS-2B cells in cell culture, and the conditioned culture medium of these cells increased ASMC proliferation in indirect co-culture experiments [93]. As a result, these findings imply that various exogenous factors and stimuli, including cigarette smoke, house dust mites (HDM), and environmental pollutants, can have an impact on ASMCs. These factors could potentially play a role in exacerbating respiratory inflammatory diseases. Therefore, it is imperative to consider not only endogenous factors, but also environmental exposures and external stimuli when investigating the etiology and pathogenesis of chronic lung conditions. Such an approach would provide a more comprehensive understanding of the complex interplay between internal and external factors that contribute to the development and progression of respiratory diseases.

## 4 Therapeutic implications of bronchial epithelial and airway smooth muscle interactions

The number of studies linking IL-8 and IL-6 to an augmentation in ASMC proliferation within models of epithelial cell injury is steadily increasing. Given that IL-8 is also strongly associated with an increase in ASMC migration in such contexts, there is a growing interest in exploring pharmacological targeting of this cytokine or its receptors as a potential leading therapeutic approach to prevent irreversible bronchial remodeling in numerous patients with COPD and asthma. Moreover, since epithelial cells play a pivotal role in initiating this remodeling process, localized application of these potential therapeutic agents via inhalers may be anticipated to yield maximal efficacy with minimal adverse effects on the immune system, in comparison to currently utilized medications. Nevertheless, we still require further research to comprehend the mechanisms by which external and internal stimuli modify airway epithelial cells, initiating their impact on bronchial smooth muscle cells. Such research could advance our treatment of chronic lung diseases with agents that act on the initial stages of the disease cascades and loops. Table 1 presents a comprehensive summary of research endeavors dedicated to elucidating the influence of bronchial epithelial cells on airway smooth muscle cells. Simultaneously, Fig. 3 illustrates the promising pathways that can be targeted to modulate interactions between BECs and ASMCs, thereby offering potential therapeutic avenues for managing chronic respiratory diseases.

**Table 1:** Summary of the research focused on understanding the impact of BECs on ASMCs.

Outcome	Model	Animals	Cell type	Stressor	Means of interaction	Mechanism	Reference
Relaxation	*In vitro*	Human Guinea Pig	BEC	None	GABA	*Unknown*	[59]
	*In vitro*	Human	BEAS-2B ASMC	None	Acetylcholine Nitric oxide	Unknown	[64]
	*In vitro*	Human	ASMC BEAS-2B BEC	None	ASMCs COX-1 Prostaglandin E receptors 2 and 4	Unknown	[67]
Contraction	*In vitro*	Human	ASMC BEC	Mechanical pressure	Endothelin-1	Unknown	[68]
	*Ex vivo/In vitro*	Rat Human	BEC	Physical injury	Unknown soluble mediators	*Unknown*	[69]
	*Ex vivo/In vitro*	Human	ASMC	Rhinovirus	IP-10 MIP-1b	Unknown	[75]
	*In vivo*	Mouse	NA	IL-13	Unknown	Unknown	[76]
	*In vivo/In vitro*	Mouse Human	BEC	IL-13	CCL2/CCL24 CXCL1	Β-arrestin pathway	[77]
	*In vivo/Ex vivo*	Mouse Human	NA	Genetic	Neuropeptide Y	*Unknown*	[55]
Migration	*In vitro*	Human	BEAS-2B BEC ASMC	YKL-40	IL-8	Activating MAPK and NF-κB Pathways	[81]
	*In vitro*	Human	ASMC BEC BEAS-2B	TNFα	IL-8 RANTES	Unknown	[79]
	*In vitro*	Human	ASMC BEC	TNFα	IL-8 CCL5	Unknown	[104]
	*In vitro*	Human	ASMC A549	CSE	IL-8 TGF-β1	M3 mAChR	[92]
	*In vitro*	Human	ASMC BEAS-2B HBE135	Nonylphenol	IL-6/IL-8	Unknown	[93]
	*In vitro*	Human	ASMC BEC	Rhinovirus	CXCL8 CCL5	Unknown	[94]
	*In vitro*	Human	ASMC BEC	Rhinovirus	CXCL10	Unknown	[95]
Proliferation	*In vitro*	Human	ASMC BEC BEAS-2B	None	ASMCs COX-1 Prostaglandin E receptors 2 and 4	*Unknown*	[67]
	*In vitro/In vivo*	Human Rabbit	ASMC BEC	Physical injury	IL-6/IL-8 MCP-1 MMP-9	*Unknown*	[54]
	*In vitro*	Human	ASMC BEC	Mechanical pressure	Endothelin-1	*Unknown*	[68]
	*In vitro*	Human	BEAS-2B BEC ASMC	YKL-40	IL-8	Activating MAPK and NF-κB Pathways	[81]
	*In vitro*	Human	ASMC BEC	Amphiregulin	Unknown	COX-2 activity in BEC	[8]
	*In vitro*	Human	ASMC 293LT1 A549 BEC	Leukotriene D4 LTD4	TGF-B1	CysLT1 receptor	[100]
	*In vitro/Ex vivo*	Human	ASMC BEC	HDM	Leukotriene C4	PAR-2 receptor	[103]
	*In vitro*	Human	ASMC BEAS-2B HBE135	Nonylphenol	IL-6/IL-8	Unknown	[93]

* BEC: Primary bronchial epithelial cell, ASMC: Primary airway smooth muscle cell, NA: Non-applicable.

**Fig. 3:** Potential Interaction pathways Between Bronchial Epithelial Cells and Airway Smooth Muscle Cells.

## 5 Conclusion

The interaction between bronchial epithelial and airway smooth muscle cells holds promise for the development of innovative therapeutic approaches for chronic lung diseases. The epithelium plays a significant role in influencing ASMC contractility, migration, and proliferation, making it a potent initiator of airway remodeling. Moreover, the effects of all stress, compression, and injury on the epithelium exacerbate this influence, thereby making the epithelium a prime suspect in inducing a vicious cycle of continuous remodeling in the airway wall. It is crucial to comprehend the impact of airway smooth muscle cells on the epithelium since manipulating these effects forms the basis for developing advanced experimental 3D models. These 3D models are increasingly gaining popularity for enhancing the credibility of *in vitro* studies by utilizing human cells in a 3D structure that closely mimics the tissue microenvironment. Such models can provide a better understanding of the complex interactions between the epithelium and ASMCs, leading to the identification of novel therapeutic targets for chronic lung diseases.

## Author contribution statement

All authors listed have significantly contributed to the development and the writing of this article.

## Funding statement

This work received no specific funding or grant.

## Data availability statement

No data was used for the research described in the article.

## Declaration of competing interest

The authors declare that they have no known competing financial interests or personal relationships that could have appeared to influence the work reported in this paper.
